The article "Left ventricular remodeling with preserved function after coronary microembolization: the effect of methylprednisolone" was published in 2014. Journal: Eur J Med Res.

# Left ventricular remodeling with preserved function after coronary microembolization: the effect of methylprednisolone

**DOI:** 10.1186/2047-783X-19-7

**Published:** 2014-02-04

**Authors:** Jianying Ma, Juying Qian, Shufu Chang, Zhangwei Chen, Hang Jin, Mengsu Zeng, Yunzeng Zou, Junbo Ge

**Affiliations:** 1 Department of Cardiology, Zhongshan Hospital, Fudan University, Shanghai 200032, China; 2 Shanghai Institute of Cardiovascular Diseases, Shanghai 200032, China; 3 Department of Radiology, Zhongshan Hospital, Fudan University, Shanghai 200032, China

**Keywords:** Coronary artery, Microembolization, Magnetic resonance imaging, Left ventricular ejection fraction, Methylprednisolone

## Abstract

**Background:**

The objective of this study was to evaluate changes in left ventricular ejection fraction (LVEF) and left ventricular remodeling after coronary microembolization (CME) and to investigate the protective effects of methylprednisolone (MTP).

**Methods:**

CME was induced by injection of microspheres (42 μm Dynospheres) into left anterior descending artery of mini swine. The animals were divided into two groups. Group 1 (*n* = 9) received 120,000 microspheres and Group 2 (*n* = 7) received 120,000 microspheres following intravenous administration of 30 mg/kg MTP. Contrast-enhanced magnetic resonance imaging (CeMRI) was performed at baseline, 6 h after intervention, and 1 week later.

**Results:**

In Group 1, LVEF was significantly decreased at 6 h but recovered 1 week. This was accompanied by continuing left ventricular remodeling. In Group 2, LVEF remained unchanged at all assessment times. LVEF measured at 6 h and 1 week after CME in Group 1 and Group 2 was 0.39 ± 0.06 and 0.44 ± 0.04, and 0.44 ± 0.04 and 0.48 ± 0.03, respectively (Both *P* >0.05). Hyperenchancement at the anterior wall of the left ventricle was shown by MRI at 6 h in Group 1 but not in Group 2. The hyperenhanced area in Group 1 was 7.77 ± 1.49% of left ventricular mass.

**Conclusions:**

The consequence of CME is left ventricular dilation with preserved LVEF. Pretreatment with MTP appears to have a cardioprotective effect on left ventricular remodeling.

## Background

Coronary microembolization (CME) can potentially lead to a perfusion-contraction mismatch, inflammation, and regional myocardial contractile dysfunction in the absence of coronary artery stenosis [1-7]. It is well recognized that left ventricular ejection fraction (LVEF) decreases during the acute phase following CME and recovers 1 week later [4,8,9]. However, previous studies with contrast-enhanced magnetic resonance imaging (CeMRI) have shown that microinfarction and left ventricular remodeling are well defined consequences of CME [8-11]. Assessment of left ventricular function using MRI is generally considered to be highly accurate and the current gold standard for calculating ventricular volumetric parameters [12,13].

Glucocorticoids have been used in various diseases to prevent or minimize inflammation [14], but controversy exists concerning the use of glucocorticoids during acute myocardial infarction [15]. To date only one study has assessed the effect of glucocorticoids after microembolization [4]. The study suggested that progressive myocardial dysfunction can be prevented by intravenous injection of methylprednisolone (MTP) prior to the onset of CME [4]. The researchers proposed that MTP decreased the inflammatory reaction caused by microinfarction [4]. In the present study, we further assessed changes in left ventricular function after CME and the effect of MTP pretreated before CME using CeMRI in an animal model developed by our team.

## Methods

### CME methodology

Sixteen mini swine of either sex (20 to 25 kg body weight) were sedated with intramuscular ketamine (5 to 10 mg/kg) and diazepam (5 to 10 mg/kg). Anesthesia was maintained with 3% pentobarbital sodium intravenously (3 mg/kg/h) until the experiment was completed.

The right femoral artery and vein were dissected and 7 F and 6 F vascular sheaths were placed in each vessel, respectively. Prior to coronary cannulation, animals were anticoagulated with intravenous heparin (5,000 IU bolus followed by 100 IU/kg/h). For coronary angiography, a 6 F XB 3.5 guiding catheter was used for the left coronary artery system via the femoral approach. A 2.8 F infusion catheter (Cordis Inc., Johnson & Johnson) was then placed in the left anterior descending (LAD) artery between the second and third diagonal branches. Microembolization was induced by continuous injection of 120,000 microspheres (42 μm Dynospheres; Dyno Particles; Lillestrøm, Norway) into the LAD followed by a 6 mL saline flush. Animals in Group 2 (*n* = 7) received 30 mg/kg MTP (in 10 mL 0.9% NaCl solution) injected intravenously 30 min before preparation for surgery. Animals in Group 1 (*n* = 9) received no MTP.

Systemic hemodynamics parameters and myocardial function were measured at baseline, 6 h, and 1 week after CME. Aortic pressure was monitored through the guiding catheter.

All animals were observed until they were awake and breathing spontaneously without intubation. The swine were anesthetized a second time 1 week later.

The experimental protocol was approved by the Animal Care and Use Committee of Fudan University, China. The animals were handled according to the guidelines of the American Physiological Society.

### Methods for MRI

MRI was performed at baseline, 6 h, and 1 week after CME using 1.5 T Magnetom (Erlangen, Siemens AG, Germany). Transverse, two-chamber, and four-chamber left ventricular long-axis scout images were obtained to determine the final short-axis image plane. Cine MR images were acquired in contiguous short-axis planes from the apex to the base of the heart to measure left ventricular function. After the cine MR images were obtained, the animals received an intravenous bolus of 0.20 mmol/kg Gd-DTPA (Magnevist; Schering, Berlin, German) at a rate of 4 mL/s by means of an infusion pump. This was followed by a 10 mL flush of saline at a rate of 4 mL/s. After 10 min, delayed images were acquired using a Turbo_flash_T1WI_PSIR_segmented sequence. The inversion time was determined at 10 min with TI-Scout sequence. Results were analyzed at Siemens Syngo Leonardo workstation [8].

### Statistical analysis

Statistical analysis was undertaken using SPSS version 11.0 software. Data were presented as means and standard deviations (±SD). Within group changes in hemodynamics (left ventricular ejection fraction (LVEF), left ventricular end diastolic volume (LVEDV), and left ventricular end systolic volume (LVESV)) were compared using a general linear model of variance for repeated measures. Independent *t* test were used to compare LVEF, LVEDV, and LVESV between groups. Values of *P* <0.05 were considered statistically significant.

## Results

Coronary thrombolysis in myocardial infarction (TIMI) grade 3 coronary flow was maintained immediately after microembolization and hemodynamic parameters remained stable before and after CME.

In Group 1, LVEF decreased at 6 h (*P* <0.01) and returned to baseline 1 week after CME. In addition LVEDV and LVESV were higher 1 week than at baseline in this group (*P* <0.01). In Group 2, there was no significant change in LVEF, LVEDV, and LVESV before or after CME. There was no difference in LVEF, LVEDV, or LVESV at 6 h between Group 1 and Group 2 (*P* = 0.08 for LVEF). However, at 1 week before and after changes in LVEDV and LVESV were significantly lower in Group 2 than in Group 1 (*P* <0.01). Before and after changes in LVEF at 6 h were significantly lower in Group 2 than in Group 1 (*P* <0.01). The results are shown in Table 1 and in Figures 1 and 2.

**Figure 1:** **Comparsion of LVEF, LVEDV, and LVESV between Groups 1 and 2.** **Compared with Group 1, *P* <0.01. Group 1: coronary microembolization with 120,000 microspheres. Group 2: coronary microembolization with 120,000 microspheres and pretreatment with methylprednisolone. LVEF: left ventricular ejection fraction; LVEDV: left ventricular end diastolic volume. LVESV: left ventricular end systolic volume.

**Figure 2:** **Before and after changes in left ventricular function between Groups 1 and 2.** **Compared with Group 1, *P* <0.01. Group 1: coronary microembolization with 120,000 microspheres. Group 2: coronary microembolization with 120,000 microspheres and pretreatment with methylprednisolone. (Δ LVEF = 6 h LVEF-baseline LVEF, ΔΔ LVEF = 1 week LVEF-baseline LVEF; Δ LVEDV = 6 h LVEDV-baseline LVEDV, ΔΔ LVEDV = 1 week LVEDV-baseline LVEDV; Δ LVESV = 6 h LVESV-baseline LVESV, ΔΔ LVESV = 1 week LVESV-baseline LVESV). LVEF: left ventricular ejection fraction; LVEDV: left ventricular end diastolic volume. LVESV: left ventricular end systolic volume. Before and after changes in LVEF at 6 h were significantly lower in Group 2 than in Group 1. At 1 week before and after changes in LVEDV and LVESV were significantly lower in Group 2 than in Group 1.

**Table 1:** Changes in LVEF, LVEDV, and LVESV in Groups 1 and 2 before and after CME

	***Baseline***	***6 h***	***One week***
LVEF			
Group 1	0.48 ± 0.06	0.39 ± 0.06^a^	0.46 ± 0.05
Group 2	0.47 ± 0.04	0.44 ± 0.04	0.48 ± 0.03
LVEDV (mL)			
Group 1	40.4 ± 3.1	40.8 ± 3.0	48.5 ± 4.0^a^
Group 2	38.0 ± 4.7	39.0 ± 6.6	37.4 ± 5.4
LVESV (mL)			
Group 1	21.0 ± 1.9	24.7 ± 1.8	26.2 ± 3.2^a^
Group 2	20.2 ± 2.4	21.8 ± 3.4	19.4 ± 2.3

Group 1: coronary microembolization with 120,000 microspheres.

Group 2: coronary microembolization with 120,000 microspheres and pretreatment with methylprednisolone.

LVEF: left ventricular ejection fraction; LVEDV: left ventricular end dilatolic volume; LVESV: left ventricular systolic volume.

^a^Compared with baseline *P* <0.01.

Hyperenchancement at anterior wall of left ventricle was apparent on CeMRI 6 h after CME in Group 1 but not in Group 2. The hyperenhanced zone was clearly visible at the anterior myocardium from the papillary to apical level (Figure 3). The area of hyperenhancment in Group 1 was 7.77 ± 1.49% of the left ventricular mass.

**Figure 3:** **Changes in CeMRI before and after CME in Group 1 and Group 2.** Group 1: coronary microembolization with 120,000 microspheres. Group 2: coronary microembolization with 120,000 microspheres and pretreatment with methylprednisolone. Hyperenhancement was demonstrated at 6 h following CME in Group 1 (white arrow) but not in Group 2. One week after CME there was no evidence of hyperenhancement on CeMRI in Group 1.

## Discussion

CME is a frequent phenomenon in patients with coronary heart disease and is particularly prevalent in patients with acute coronary syndrome (ACS). It is a marker for fatal events, especially in patients undergoing percutaneous coronary intervention (PCI) [16-19]. Rupture of the atherosclerotic plaque in the epicardial coronary artery is the main cause of CME in clinical practice [18]. The consequence of CME may also be related fatal events in patients with unstable angina pectoris [17,18].

In the present study, we addressed changes in left ventricular function after CME and investigated the possible protective role of methylprednisolone. Our objective was to better understand the development of CME and to evaluate the possible benefit of glucocorticoid pretreatment. Using an experimental model developed by our team, we demonstrated impairment of left ventricular function (evidenced by changes in LVEF) at 6 h, recovers spontaneously 1 week later after CME, but left ventricular remodeling continues [8]. We also showed that pretreatment with MTP before CME may prevent the progression of remodeling.

Based on these findings, the observed changes were thought to be related to an inflammatory response rather than to micro-infarction after CME. Previous studies have demonstrated that myocardial infarction following CME affects only about 2% to 5% of the perfusion territory, and that apoptosis is almost negligible [1,5]. Our results supported these findings as hyperenhancement 6 h after CME accounted for no more that 8% of left ventricular mass.

Previous studies have shown that inflammatory responses induced by microinfarction, is mediated by monocytes, macrophage infiltration, and the release of inflammatory factors [2,8]. In a previous study we showed that the degree of inflammation was markedly higher in the embolized zone than that in the control zone [9]. We also demonstrated that increased serum MCP-1 promotes leukocyte infiltration and that this is followed by a classical inflammatory response [9], suggesting that inflammation and oxygen-free radicals are involved in left ventricular remodeling [5,9,20-23].

In our experiments LVEF was preserved 1 week after CME due to left ventricular remodeling, which occurred as a consequence of the persistent inflammatory response in the embolized zone. A previous study, using MRI to evaluate changes after CME, demonstrated a significant decline in LVEF 1 h and 1 week after intervention [11]. The difference between these findings and our own may be related to differences in the sizes of microspheres used in the animal models. Thus, it is possible that larger diameter microspheres might result in a more persistent decline in LVEF.

In our previous study, hyperenchancement was observed 6 h after CME [8]. This hyperenhancement was disappeared 1 week later without any treatment. The reason for this may be related to the presence of acute myocardial microinfarction and acute myocardial edema 6 h after CME. However, after 1 week, the myocardial edema would have disappeared and the spatial resolution of MRI may not have been high enough to detect the experimentally induced microinfarcts.

An important finding of the present study was that pretreatment with MTP eliminated the hyperenhancement at 6 h after CME and protected the decline of LVEF as well as left ventricular remodeling. The anti-inflammatory effects of glucocorticoids have been widely used for the treatment of a variety of diseases in clinical practice. In experimental studies, glucocorticoids have been shown to attenuate the interaction of leukocytes with endothelium [24] and to inhibit the infiltration of macrophages/monocytes [25]. Glucocorticoid-induced suppression of the generation and release of inflammatory cytokines and mediators have also been demonstrated [25,26]. However, the effects of glucocorticoids in the treatment of acute myocardial infarction remained controversial [27].

A previous study reported that MTP was able to protect against progressive myocardial contractile dysfunction after CME, suggested that it may have a cardioprotective effect in this setting [4]. These findings are supported by the results of the present study and suggest that pretreatment with MTP inhibits the inflammatory response and attenuates myocardial edema induced by CME [4]. This effect was also reflected by the absence of delayed hyperenhancement 6 h after CME in the pretreated group. As a result of the reduced levels of the inflammation, LVEF remained unchanged and left ventricular remodeling was no longer present 1 week after CME. These results suggest that pretreatment with glucocorticoids may prevent left ventricular remodeling after CME in the clinical practice [4]. However further studies are needed to substantiate these findings.

As there was no control group in our study it was not possible to eliminate changes due to the surgical procedure. However, previous studies have demonstrated this type of animal model closely resembles CME seen in clinical practice and in previous studies control groups were not used. A second limitation is that this animal model resembles but does not exactly replicate the sequence of events that occurs following complications of percutaneous coronary intervention. In clinical practice the thromboemboli are frequently much larger, are of non-uniform diameter, and do not always result in myocardial damage. In future studies, a longer observation period should be adopted to observe the long-term effects of CME and glucorcoticoids on left ventricular remodeling.

## Conclusions

Our results demonstrate that experimentally induced CME resulted in left ventricular dilation with preserved LVEF. Pretreatment with MTP had a cardioprotective effect on left ventricular remodeling. These findings are of potential significance for the clinical management of CME.

## Abbreviations

ACS: Acute coronary syndrome; CeMRI: Contrast enhanced magnetic resonance imaging; CME: Coronary microembolization; LAD: Left anterior descending; LVEDV: Left ventricular end diastolic volume; LVEF: Left ventricular ejection fraction; LVESV: Left ventricular end systolic volume; MTP: Methylprednisolone; PCI: Percutaneous coronary intervention; TIMI: Thrombolysis in myocardial infarction.

## Competing interests

The authors have no competing interests.

## Authors' contributions

JM carried out the animal studies, performed the statistical analysis, and drafted the manuscript. JQ participated in the design of the study and helped to draft the manuscript. SC participated in the animal model preparation and construction. ZC participated in the animal model construction. HJ participated in the MRI and data collection. MZ participated in the MRI. YZ participated in the design of the study and helped to perform the statistical analysis. JG conceived of the study, and participated in its design and helped to draft the manuscript. All authors read and approved the final manuscript.

## Authors' information

Jianying Ma: PhD, MD, Associate Professor of Medicine/Cardiology, Department of Cardiology, Zhongshan hospital, Fudan University; Shanghai institute of Cardiovascular disease, Shanghai, China. Juying Qian: MD, FSCAI, Professor of Medicine/Cardiology, Deputy Director of Department of Cardiology, Zhongshan hospital, Fudan University; Shanghai institute of Cardiovascular disease, Shanghai, China. Shufu Chang: MD, Attending physician, Department of Cardiology, Zhongshan hospital, Fudan University; Shanghai institute of Cardiovascular disease, Shanghai, China. Zhangwei Chen: MD, Attending physician, Department of Cardiology, Zhongshan hospital, Fudan University; Shanghai institute of Cardiovascular disease, Shanghai, China, Shanghai, China. Hang Jin: PhD, MD, Associate professor of Radiology, Department of Radiology, Zhongshan hospital, Fudan University, Shanghai, China. Mengsu Zeng: PhD, MD, Professor of Radiology, Director of Department of Radiology, Zhongshan hospital, Fudan University, Shanghai, China. Yunzeng Zou: Professor of Institute of Biomedical Science; Professor of Medicine/Cardiology, Department of Cardiology, Zhongshan hospital, Fudan University; Shanghai institute of Cardiovascular disease, Shanghai, China. GE Junbo, MD, FESC, FACC, FSCAI, Professor of Medicine/Cardiology, Director of Department of Cardiology, Zhongshan Hospital, Fudan University; Director of Shanghai Institute of Cardiovascular Diseases, Shanghai, China.
